This article has been retracted.

# Tripterine up-regulates miR-223 to alleviate lipopolysaccharide-induced damage in murine chondrogenic ATDC5 cells

**DOI:** 10.1177/2058738418824521

**Published:** 2019-01-18

**Authors:** Xuefu Li, Wei Wei, Zhongquan Zhao, Shuzhen Lv

**Affiliations:** Department of Orthopedics, Liaocheng Third People’s Hospital, Liaocheng, China

**Keywords:** ATDC5 cell, lipopolysaccharides, miR-223, osteoarthritis, tripterine

## Abstract

Tripterine, also known as celastrol, is a main natural ingredient in *Tripterygium wilfordii*. Tripterine has a variety of pharmacological functions, and the therapeutic potential of tripterine in many kinds of inflammation-linked diseases has been revealed. However, the function of tripterine on osteoarthritis still remains unclear. The objective of this study was to study the function of tripterine (TPR) on lipopolysaccharide (LPS)-injured chondrocyte. ATDC5 cells were treated with tripterine after LPS stimulation and then cell survival, the release of pro-inflammatory cytokines, and the expression of chondrogenic differentiation-associated proteins were assessed by performing CCK-8, flow cytometry, reverse transcription quantitative polymerase chain reaction (RT-qPCR), enzyme-linked immunosorbent assay (ELISA), and Western blot. Moreover, the expression of miR-223 and core factors in PI3K/AKT and nuclear factor kappa B (NF-κB) signaling was tested by RT-qPCR/Western blot. LPS stimulation significantly reduced ATDC5 cells viability, induced apoptosis, and increased the release of interleukin (IL)-6 and tumor necrosis factor (TNF)-α. Tripterine protected ATDC5 cells against LPS-induced chondrocyte loss and the release of IL-6 and TNF-α. miR-223 was down-regulated by LPS, while was up-regulated by tripterine. The protective actions of tripterine were eliminated when miR-223 was silenced. Besides, tripterine inhibited hypertrophic differentiation induced by LPS, and the inhibitory effects of tripterine on hypertrophic differentiation could be abolished when miR-223 was silenced. Furthermore, tripterine activated PI3K/AKT pathway and deactivated NF-κB pathway. And the regulatory effects of tripterine on these two pathways were abolished by miR-223 silence. This study revealed that tripterine protected ATDC5 cells against LPS-induced cell damage possibly via up-regulation of miR-223 and modulation of NF-κB and PI3K/AKT pathways.

## Introduction

Osteoarthritis is a common degenerative disease among elderly.^1^ It causes severe pain and joint movement disorders.^2^ What’s worse, the pain will make it difficult to exercise and results in muscle loss.^3^ Multiple factors have been found to be involved in the pathogenesis of osteoarthritis, including age, obesity, trauma, congenital anomaly of joint, joint deformity, and so on. However, the detailed pathogenesis of osteoarthritis remains unclear. Treatment of osteoarthritis depends on symptomatology. For overweight patients, lifestyle change is one of the treatment options.^4^ For others, medication is recommended, but this option is limited in the management of pain. Joint replacement surgery is another main treatment for the patients, whose quality of life is significantly reduced by osteoarthritis. However, there are problems getting the repair of cartilaginous lesions within synovial joints.^5^ These facts call for a more effective treatment strategy for osteoarthritis.

Tripterine, also known as celastrol, is a natural compound mainly isolated from traditional Chinese medicine herb *Tripterygium wilfordii*. It is a pentacyclic triterpene with a variety of bioactivities. Tripterine has been found to have anti-inflammatory,^6^ anti-tumor,^7,8^ antioxidant,^9^ anti-fibrotic,^10^ and anti-obesity^11^ activities. In clinic, tripterine is used to treat rheumatoid arthritis, leprosy reaction, as well as other autoimmune diseases such as systemic lupus erythematosus.^12,13^ Besides, it has been revealed that tripterine modulates cell survival and inflammation via regulation of nuclear factor kappa B (NF-κB), MAPK, JAK/STAT, and PI3K/AKT pathways.^12,13^ And also, an in vitro study demonstrated that triterpene treatment was capable of decreasing the expression of matrix metalloproteinase (MMP)-1, MMP-3, MMP-13, inducible nitric oxide synthase 2 (iNOS-2), and cyclooxygenase-2 (COX-2), suggesting tripterine as a potential agent for the treatment of osteo-arthritis.^14^ However, the anti-osteoarthritis effects of tripterine have not been studied well, and the mechanism of action is still a mystery.

microRNAs (miRNAs) are a kind of endogenous, short (with about 18–25 nucleotides), and highly conserved non-coding RNAs. miRNAs provide robustness to gene regulation, and they contribute to a wide range of pathologies, including chronic inflammation.^15^ In patients with osteoarthritis and rheumatoid arthritis, miR-223 of synovial fluid was significantly down-regulated.^16^ Besides, the up-regulation of miR-223 in peripheral blood mononuclear cells of osteoarthritis is related with healthy subjects, as early stages of osteoarthritis possessed a higher miR-223 level than the later stages.^17^ Aziz^18^ has mentioned miR-223 as a novel potential diagnostic and therapeutic target for inflammatory disorders. All together, these authors proposed miR-223 as an osteoarthritis-associated miRNA.

ATDC5 is a chondrogenic cell line derived from a differentiating culture of AT805 teratocarcinoma cells, which has been considered as an excellent in vitro model cell line for chondrogenesis.^19^ It has properties to reproduce multi-steps of chondrocyte differentiation, and can easily proliferate so that vast amounts of cells can be obtained to set up in vitro culture system, and can mimic the cellular condensation during chondrogenesis. This study assessed the function of tripterine in lipopolysaccharide (LPS)-injured ATDC5 cells, in order to reveal the potential of tripterine in the treatment of osteoarthritis in vitro. In addition, the regulatory effect of tripterine on miR-223 expression was tested to decode the underlying mechanisms of which tripterine protected ATDC5 cells against LPS.

## Materials and methods

### Cell culture

ATDC5 cells purchased from the European Collection of Authenticated Cell Cultures (ECACC, Salisbury, UK) were cultured in DMEM: Ham’s F12 (1:1) (Sigma-Aldrich, St Louis, MO, USA), plus 2 mM Glutamine (Gibco, Grand Island, NY, USA), and 5% fetal bovine serum (FBS, Gibco). The cells were maintained at 37°C in a humidified incubator containing 5% CO_2_. Subcultures were obtained using 0.25% trypsin/EDTA solution (Sigma-Aldrich) every 3 days.

LPS from *Escherichia coli* O111:B4 was purchased from Sigma-Aldrich. The cells were treated with various doses of LPS for 12 h.

Tripterine with purity greater than 98% was purchased from Sigma-Aldrich. Tripterine was dissolved in dimethyl sulfoxide (DMSO; Sigma-Aldrich) and made up with the culture medium so that the concentration of DMSO was 0.1%. The cells were treated with various doses of tripterine for 4 h after LPS stimulation. The cells treated with 0.1% DMSO were used as negative control (NC).

For cell differentiation, ATDC5 cells were cultured as above mentioned for 14 days. Hypertrophic differentiation was induced by addition of 10 g/mL insulin, 10 g/mL transferrin, and 10 g/mL selenium (all from Sigma-Aldrich) for another 14 days. Each medium was replaced every 3 days.

### Cell viability assessment

ATDC5 cells were seeded in 96-well plates with a density of 5 × 10^3^ cells/well. After adhesion, the cells were treated with LPS with or without tripterine and then the culture medium was removed, and 10 μL CCK-8 solution (Dojindo Molecular Technologies, Kyushu, Japan) was added into each well. The plates were cultured at 37°C in a humidified incubator for 4 h. The absorbance of each well was measured at 450 nm using a Microplate Reader (Bio-Rad, Hercules, CA, USA).

### Quantitation of apoptosis

ATDC5 cells were seeded in six-well plates with a density of 5 × 10^5^ cells/well. After adhesion, the cells were treated with LPS with or without tripterine, after which the apoptosis was detected using Annexin V-fluorescein isothiocyanate (FITC)/propidium iodide (PI) apoptosis detection kit (Beijing Biosea Biotechnology, Beijing, China). The cells were collected using the trypsin solution (Sigma-Aldrich). At least 1 × 10^5^ cells of each sample were resuspended in 200 μL binding buffer, containing 5 μL of Annexin V-FITC and 10 μL of PI. The samples were then incubated in the dark at room temperature for 30 min. Then, 300 μL of phosphate-buffered saline (PBS) was added into the sample, and the apoptosis analysis was done by a flow cytometer (Beckman Coulter, USA). The rate of apoptotic cells (Annexin-V positive and PI-negative) was analyzed by the FCS Express software (De Novo software, Los Angeles, CA, USA).

### Enzyme-linked immunosorbent assay

ATDC5 cells were seeded in 24-well plates with a density of 5 × 10^4^ cells/well. The cells were treated with LPS with or without tripterine, after which the culture supernatant was collected. The concentrations of pro-inflammatory cytokines, including interleukin (IL)-6 and tumor necrosis factor (TNF)-α, were measured using the corresponding enzyme-linked immunosorbent assay (ELISA) kits (R&D Systems, Abingdon, UK).

### miRNAs transfection

The pre-miR-223, anti-miR-223, and the NC were synthesized by GenePharma Co. (Shanghai, China). Cell transfection was performed using the Lipo-fectamine 3000 reagent (Invitrogen, Carlsbad, CA, USA). At 48 h of transfection, cells were collected for use in the following experiments.

### Reverse transcription quantitative polymerase chain reaction (RT-qPCR)

Total RNA was isolated from ATDC5 cells using TRIzol reagent (Invitrogen). Reverse transcription was performed using 1 μg of total RNA and the PrimeScript Reverse Transcriptase (Takara, Dalian, China). RT-qPCR was performed by Taqman Universal Master Mix II (Applied Biosystems, Foster City, CA). β-actin served as an internal control for IL-6, TNF-α, Collagen X, and MMP-13. U6 snRNA served as an internal control for miR-223. Data were calculated according to the 2^-ΔΔCt^ method.

### Western blot

Cellular protein was extracted using the RIA lysis buffer (Beyotime Biotechnology, Shanghai, China). The purity of the extracts was tested by BCA™ Protein Assay Kit (Pierce, Appleton, WI, USA). Proteins were separated by the sodium dodecyl sulfate polyacrylamide gel electrophoresis (SDS-PAGE) and were transferred onto polyvinylidene difluoride (PVDF) membranes (Millipore, MA, USA). After blocking with 5% non-fat milk for 1 h, the membranes were probed by the antibodies at 4°C overnight, for the detection of Bcl-2 (ab692), Bax (ab77566), pro-caspase-3 (ab4051), cleaved-caspase-3 (ab13847), IL-6 (ab6672), TNF-α (ab6671), PI3K (ab191606), p-PI3K (ab182651), AKT (ab8805), p-AKT (ab38449), IκBα (ab32518), p-IκBα (ab133462), p65 (ab16502), p-p65 (ab86299), Collagen II (ab188570), Aggrecan (ab3778), MMP-3 (ab53015), MMP-13 (ab51072), and β-actin (ab8226, Abcam, Cambridge, MA, USA). The membranes were then incubated with the secondary antibodies for 1 h at room temperature. Signals were developed using ECL Plus Western Blotting Substrate (Pierce, Carlsbad, CA, USA). The intensity of the bands was quantified using Image Lab™ Software (Bio-Rad, Shanghai, China).

### Statistical analysis

All the experiments were repeated three times. Results were presented as the mean ± standard deviation (SD). Statistical analyses were performed using SPSS 19.0 statistical software (SPSS Inc., Chicago, IL, USA). The *P*-values were calculated using one-way analysis of variance (ANOVA) or Student’s *t* test. A *P*-value of <0.05 was considered to indicate a statistically significant result.

## Results

### LPS-induced cell damage in ATDC5 cells

To start with, ATDC5 cells were treated with various doses of LPS for 12 h. CCK-8 assay results in Figure 1(a) indicate that LPS damaged ATDC5 cells viability in a dose-dependent manner. Considering 8 μg/mL LPS-induced cell viability reduction of 50.69% (*P* < 0.01), 8 μg/mL was selected as a LPS-stimulating condition for use in the following experiments. Figure 1(b) shows that apoptosis rate was significantly increased in LPS group than that in the control group (*P* < 0.01). Consistently, Western blot analytical results displayed that Bcl-2 was down-regulated, Bax was up-regulated, and caspase-3 was cleaved remarkably in LPS group than those in the control group (Figure 1(c)).

**Figure 1.** LPS-induced cell damage in ATDC5 cells. (a) The viability of ATDC5 cells was measured after treating with various doses of LPS. (b) Apoptosis rate, (c) expression of apoptosis-related proteins, (d) mRNA levels of IL-6 and TNF-α, (e) protein levels of IL-6 and TNF-α, and (f) concentrations of IL-6 and TNF-α in culture supernatant were respectively assessed following 8 μg/mL LPS stimulation. *P < 0.05, **P < 0.01, and ***P < 0.001.

Next, the expression changes of pro-inflammatory cytokines, including IL-6 and TNF-α, following LPS stimulation were tested. As results shown in Figure 1(d) and (e), both the messenger RNA (mRNA; *P* < 0.01 and *P* < 0.001) and protein levels of IL-6 and TNF-α were higher in LPS group when compared to the control group. And also, the concentrations of IL-6 and TNF-α in the culture supernatant were much higher in the LPS group when compared to the control group (both *P* < 0.001, Figure 1(f)).

### Tripterine attenuated LPS-induced cell damage

Various doses of tripterine were used to treat ATDC5 cells, and cell viability was measured to test the cytotoxicity of tripterine. Data in- Figure 2(a) show that cell viability was unaffected by tripterine treatment with concentrations equal to or less than 2 μM. But, the viability of ATDC5 cells was significantly reduced by 3 (*P* < 0.05) and 4 μM (*P* < 0.01) of tripterine. Tripterine with a final concentration of 2 μM was selected for use in the follow-up experiments. Figure 2(b)–(d) shows that the viability was increased (*P* < 0.05), apoptosis rate was decreased (*P* < 0.05), Bcl-2 was up-regulated, Bax was down-regulated, and the cleavage of caspase-3 was repressed in (LPS + TPR) group than those in the LPS group. Besides, the expression and release of IL-6 and TNF-α were decreased significantly in the LPS + TPR group as compared to the LPS group (Figure 2(e)–(g)). These data collectively suggested that cell death and the release of pro-inflammatory cytokines induced by LPS could be attenuated by tripterine treatment.

**Figure 2.** Tripterine attenuated LPS-induced cell damage. (a) The viability of ATDC5 cells was tested after various doses of tripterine treatment. (b) The viability of ATDC5 cells, (c) apoptosis rate, (d) expression of apoptosis-related proteins, (e) mRNA levels of IL-6 and TNF-α, (f) protein levels of IL-6 and TNF-α, and (g) concentrations of IL-6 and TNF-α were respectively assessed following 8 μg/mL LPS treatment alone or in combination with 2 μM tripterine treatment. *P < 0.05, **P < 0.01, and ***P < 0.001.

### Tripterine elevated the expression of miR-223

miR-223 has been reported to be down-regulated in response to LPS.^20^ This phenomenon was also observed in this study. As shown in Figure 3, the expression of miR-223 was significantly reduced by LPS stimulation (*P* < 0.05). However, when compared to the LPS group, the miR-223 expression was significantly increased in the LPS + TPR group (*P* < 0.01), indicating the dysregulated miR-223 might be involved in the treating effects of tripterine on LPS-induced cell damage.

**Figure 3.** Tripterine elevated the expression of miR-223. The expression changes of miR-223 were determined in ATDC5 cells following 8 μg/mL LPS treatment alone or in combination with 2 μM tripterine treatment. *P < 0.05 and **P < 0.01.

### Tripterine attenuated LPS-induced cell damage through up-regulation of miR-223

Next, the expression levels of miR-223 in ATDC5 cells were altered by miRNA transfection. RT-qPCR data in Figure 4(a) show that the expression of miR-223 was significantly increased by pre-miR-223 transfection (*P* < 0.01) and was significantly decreased by anti-miR-223 transfection (*P* < 0.01). Figure 4(b)–(d) shows that transfection of cells with anti-miR-223 significantly decreased cell viability (*P* < 0.01), increased apoptosis (*P* < 0.05), down-regulated Bcl-2, up-regulated Bax, and cleaved caspase-3 when compared to the cells transfected with NC. Figure 4(e)–(g) shows that transfection of cells with anti-miR-223 also significantly increased the expression and release of IL-6 and TNF-α when compared to the cells transfected with NC. In contrast, pre-miR-223 transfection impacted ATDC5 cells viability, apoptosis, and the release of IL-6 and TNF-α, resulting in apposite results. These data suggested that the treating activities of tripterine on LPS-induced cell damage could be flattened by miR-223 silence.

**Figure 4.** Tripterine attenuated LPS-induced cell damage through up-regulation of miR-223. (a) The expression changes of miR-223 were determined in ATDC5 cells following miRNA transfection. (b) The viability of ATDC5 cells, (c) apoptosis rate, (d) expression of apoptosis-related proteins, (e) mRNA levels of IL-6 and TNF-α, (f) protein levels of IL-6 and TNF-α, and (g) concentrations of IL-6 and TNF-α in culture supernatant were respectively assessed following miRNA transfection and 8 μg/mL LPS treatment alone or in combination with 2 μM tripterine treatment. *P < 0.05, **P < 0.01, and ***P < 0.001.

### Tripterine inhibited hypertrophic differentiation through up-regulation of miR-223

In order to address whether endogenous miR-223 was changed during ATDC5 cells differentiation, RT-qPCR was conducted. As shown in Figure 5(a), miR-223 expression was significantly declined at the 14th day of culturing in differentiation media (*P* < 0.05), and miR-223 expression reached a minimum at the 28th day (*P* < 0.01). In addition, the mRNA levels of hypertrophic factors like Collagen X and MMP-13 were significantly up-regulated by LPS stimulation (*P* < 0.01 or *P* < 0.001) and down-regulated by addition of tripterine (*P* < 0.05 or *P* < 0.01, Figure 5(b)). These data indicated the potential roles of miR-223 and tripterine in hypertrophic differentiation. To further strengthen this hypothesis, ATDC5 cells were transfected with anti-miR-223 or pre-miR-223 in combination with tripterine treatment, and the expression changes of chondrocyte-specific markers were measured by Western blot analysis. Figure 5(c) shows that Collagen II and Aggrecan expression was remarkably down-regulated by LPS, while MMP-3 and MMP-13 expression was up-regulated. As expected, tripterine treatment partially recovered the impacts of LPS on these proteins’ expression, and the recovery effects could be attenuated by pre-miR-223 and accelerated by anti-miR-223.

**Figure 5.** Tripterine inhibited hypertrophic differentiation through up-regulation of miR-223. (a) RT-qPCR analysis for testing the expression changes of miR-223 after culturing in differentiation media for 0–28 days. (b) RT-qPCR analysis for testing the expression changes of hypertrophic factors, that is, Collagen X and MMP-13, after treating with 2 μM tripterine. (c) Western blotting for measurement of protein expression of chondrocyte-specific markers after the untransfected or transfected cells treating with 8 μg/mL LPS alone or in combination with 2 μM tripterine. *P < 0.05, **P < 0.01, and ***P < 0.001.

### Tripterine up-regulated miR-223 to activate PI3K/AKT signaling and deactivate NF-κB signaling

Finally, the expression changes of core factors in PI3K/AKT and NF-κB signaling pathways were tested by Western blot. Results in Figure 6(a)–(d) show that LPS significantly increased the phosphorylation of PI3K (*P* < 0.05), IκBα (*P* < 0.001), and p65 (*P* < 0.05). LPS slightly increased the phosphorylation of AKT, but the increase was not significant. Tripterine treatment significantly accelerated the phosphorylation of PI3K and AKT, but repressed the phosphorylation of IκBα and p65 (all *P* < 0.05). More importantly, the regulation of tripterine on these four proteins was eliminated by anti-miR-223 (*P* < 0.05 or *P* < 0.01) and was enhanced by pre-miR-223 (*P* < 0.01 or *P* < 0.001).

**Figure 6.** Tripterine up-regulated miR-223 to activate PI3K/AKT signaling and deactivate NF-κB signaling. (a, b) Protein expression changes of PI3K and AKT, as well as (c, d) IκBα and p65 were measured in ATDC5 cells following miRNA transfection and 8 μg/mL LPS treatment alone or in combination with 2 μM tripterine treatment. ns: no significance; *P < 0.05, **P < 0.01, and ***P < 0.001.

## Discussion

Osteoarthritis is a kind of noninflammatory disease. However, it has been verified that inflammatory response can contribute to the pathogenesis of osteoarthritis.^21^ IL-6 and TNF-α are two important cytokines in the physiopathogenesis of osteoarthritis. The secreted IL-6 and TNF-α increase the expression of MMPs and the amounts of NO, which in turn induce the loss of extracellular matrix and chondrocyte.^21,22^ LPS, also known as endotoxin, contributes to low-grade inflammation including the pathogenesis of osteoarthritis.^23^ LPS has been considered as a major hidden risk of osteoarthritis.^24^ In this study, LPS was used to mimic an in vitro model of osteoarthritis in ATDC5 cells. As a result, LPS stimulation significantly reduced ATDC5 cells survival and increased the release of pro-inflammatory cytokines (IL-6 and TNF-α). These data suggested that the in vitro model of osteoarthritis was established successfully. More importantly, we found that tripterine protected ATDC5 cells against LPS-induced cell damage. miR-223 was up-regulated in response to tripterine treatment, and the dysregulated miR-223 might be implicated in the protective functions of tripterine.

In China, *T. wilfordii* has been clinically used as a traditional Chinese herb for treating rheumatoid arthritis, rheumatic arthritis, nephritis, lupus erythematosus, Sjogren’s syndrome, psoriasis, scabies, and so on. In recent years, with the development of analytical techniques, tripterine has been recognized as a main natural ingredient in *T. wilfordii*, and a variety of tripterine’s pharmacological functions have been revealed. Among which, the anti-inflammatory activity of tripterine has been widely reported.^12^ A previous study has demonstrated that tripterine was capable of protecting human chondrocytes against IL-1β-induced up-regulations of MMPs, iNOS, and COX-2.^14^ Our data were consistent with this study, suggesting that tripterine protected ATDC5 cells against LPS-induced chondrocyte loss and inflammatory response, as cell viability was increased, apoptosis was inhibited, and the release of IL-6 and TNF-α was repressed.

Although the anti-inflammatory action of tripterine has been widely accepted, the underlying mechanisms are still unclear. Hu et al.^25^ have reported that tripterine conferred its anti-inflammatory effect by inducing Nur77 mitochondrial translocation. Zhang et al.^26^ suggested that tripterine exhibited its anti-inflammatory effect via mediating T helper 17 (Th17) cell/regulatory T (Treg) cell imbalance. But herein, we focused on the regulatory effect of tripterine on miRNA regulation. Actually, various miRNAs have been mentioned as targets for tripterine, including miR-101,^27^ miR-21,^28^ miR-224,^29^ miR-17-92a,^30^ and miR-223.^31^ In human breast cancer cell line and prostate cancer line, tripterine caused the elevation of miR-223, and then contributed to tripterine’s anti-cancer actions.^31^ In this study, we revealed that miR-223 level could also be elevated in ATDC5 cells. And in vitro rescue assay results suggested that tripterine reduced the apoptosis and inflammation induced by LPS might be via up-regulation of miR-223.

Apart from the cell growth-promoting and anti-inflammatory effects, the correlation between tripterine and chondrogenic differentiation was also studied in this study. By performing RT-qPCR, we found that tripterine treatment reduced the expression of hypertrophic factors like Collagen X and MMP-13. Meanwhile, miR-223 expression was found to be declined when culturing in differentiation media, suggesting miR-223 was down-regulated with the conduct of cell differentiation. What’s more, tripterine up-regulated Collagen II and Aggrecan protein expression and down-regulated MMP-3 and MMP-13 protein expression through up-regulating miR-223. These findings collectively suggested that tripterine inhibited hypertrophic differentiation through up-regulation of miR-223, which further strengthened the anti-osteoarthritis effect of tripterine. The anti-osteoarthritis activities of tripterine and the involvement of miR-223 in osteoarthritis have been previously revealed. However, this study demonstrated for the first time that tripterine conferred its anti-osteoarthritis effects via regulating miR-223.

NF-κB and PI3K/AKT pathways are central regulators of inflammation and cell survival, which can determine cell’s fate. Both of them are involved in the pathogenesis of osteoarthritis.^32,33^ Upon stimulation of cells with LPS, NF-κB pathway is activated while PI3K/AKT is deactivated, which leads to the activation of a number of cytokines, chemokines, and pro-inflammatory mediators.^34,35^ Therefore, modulation of NF-κB pathway and activating PI3K/AKT pathways can be considered as potential strategies for controlling of inflammatory responses. Moreover, tripterine could control inflammation by targeting both NF-κB and PI3K/AKT pathways.^12^ In this study, we observed that tripterine activated PI3K/AKT signaling and deactivated NF-κB signaling. In addition, the regulatory effects of tripterine on these two pathways were abolished by miR-223 silence. These data indicated that tripterine up-regulated miR-223, which in turn activated PI3K/AKT and deactivated NF-κB, and ultimately conferred protection on ATDC5 cells following LPS stimulation.

In conclusion, this study revealed that tripterine protected ATDC5 cells against LPS-induced cell loss and inflammation possibly via up-regulation of miR-223 and modulation of NF-κB and PI3K/AKT pathways. The findings of this study provided in vitro evidence that tripterine might be a potential anti-osteoarthritis agent.
